The article "A Classification Method for Thoracolumbar Vertebral Fractures due to Basketball Sports Injury Based on Deep Learning" was published in 2022. Journal: Comput Math Methods Med.

# A Classification Method for Thoracolumbar Vertebral Fractures due to Basketball Sports Injury Based on Deep Learning

**DOI:** 10.1155/2022/8747487

**Published:** 2022-10-05

**Authors:** XiaoGan Chen, Yu Liu

**Affiliations:** ^1^Wuxi Taihu University, Wuxi Jiangsu 214000, China; ^2^Wuxi 9th People's Hospital Affiliated to Soochow University, Wuxi Jiangsu 214000, China

## Abstract

**Objective:**

There are more and more basketball competitions, to propose a classification method of thoracolumbar fractures to assist in the diagnosis of basketball injuries, to analyze the feasibility of its clinical application, and to improve the recovery rate.

**Methods:**

From February 2015 to May 2022, 1130 CT images of thoracolumbar fractures admitted to our hospital and affiliated hospital units due to basketball injuries were collected, and the image labeling system uniformly labeled them. All CT images were classified according to the AO spine classification of thoracolumbar injuries. In the ABC-type classification, 935 CT images were used for training and validation to optimize the deep learning system, including 815 training sets and 120 validation sets; the remaining 198 CT images were used as test sets for comparing the deep learning system and clinician's diagnosis. In the classification of subtype A, a total of 523 CT scans can be performed for training and validation to optimize the deep learning system, including 500 training sets and 23 validation sets; the remaining 94 CT images are used as test sets for comparing depth learning systems and clinicians' diagnostic results.

**Results:**

The deep learning system had a correct rate of ABC classification of fractures in 86.4%, with a kappa coefficient of 0.850 (*P* < 0.001); the correct rate of subtype A was 85.3%, with a kappa coefficient of 0.815 (*P* < 0.001).

**Conclusion:**

The classification accuracy of thoracolumbar fractures based on deep learning is high. The method can assist in diagnosing CT images of thoracolumbar fractures and improve the current manual and complex diagnosis process.

## 1. Introduction

From the analysis of the status quo of clinical treatment of basketball injuries, basketball is a ball sport with strong collective antagonism. Offense and defense alternate instantaneously, sudden start and stop, jumping and squatting, body position changes, etc.; players constantly change. Action is a characteristic of basketball, so basketball is very prone to various sports injuries, and the incidence of fractures continues to rise. The incidence of medical disputes in fracture diagnosis remains high. Improving the timeliness, accuracy, and comprehensiveness of fracture diagnosis is necessary. Conventional radiographic diagnosis is difficult for occult or minor fractures in fracture diagnosis. Once missed or misdiagnosed, it may lead to complications such as compression plate fracture, deep infection, delayed fracture union, or nonunion. Improve fracture diagnosis techniques.

The article "A Classification Method for Thoracolumbar Vertebral Fractures due to Basketball Sports Injury Based on Deep Learning" was published in 2022. Journal: Comput Math Methods Med.

The current fracture diagnostic typing is based on simple typing of fracture morphology or neurological function score, which can only distinguish the general location, morphology, and degree of fracture. The diagnostic typing of the same patient varies greatly among clinicians. The current fracture diagnostic typing system is less intelligent and less consistent and lacks guidance on personalized treatment modalities, which is not conducive to forming and applying standardized treatment plans for spinal fractures. Therefore, a classification method is urgently needed to unify the typing and diagnose fracture types.

Deep learning technology is applied in the clinical medical field mainly for reading and diagnosing medical images. The deep learning technology can quickly mark abnormal structures or areas in the medical images of patients, providing important references for doctors' judgment and diagnosis. Current research on medical image processing based on deep learning technology is mainly focused on large [1–3], liver [4], pancreas [5], prostate [6], multiorgan [7], and fracture analysis [8–10]. Artificial intelligence diagnosis technology based on medical imaging is still in the preliminary exploration stage in the field of orthopedics [11–14]. The study of orthopedic diagnosis problems from the perspective of artificial intelligence, especially for the identification and autonomous localization of thoracolumbar vertebrae [15–19], is still in urgent need of more in-depth research. This study proposes a novel classification method for fractures based on fast-region convolutional neural network (Faster RCNN) deep learning to improve the complex manual diagnosis process.

## 2. Materials and Methods

### 2.1. Study Subjects

The CT images of all cases this time include 1130 fracture CT images collected in our hospital and affiliated hospitals from February 2015 to May 2022, which were injured in basketball and collected in our hospital and affiliated hospitals. Images of fractures were observed. As sample data, exclude unique samples with special bone structures such as severe shadow shading, hidden fractures, and osteoporosis.

### 2.2. Faster RCNN-Based Fracture Classification

This study establishes a fracture classification method based on the Faster RCNN deep learning network. For the problem of various types of fractures, the Faster RCNN is applied to iteratively learn a large number of prelabeled CT sample data of fracture types, extract the different features of various types of fracture sample data as the input of the classifier, and achieve the classification of the corresponding fracture test sample data.

The article "A Classification Method for Thoracolumbar Vertebral Fractures due to Basketball Sports Injury Based on Deep Learning" was published in 2022. Journal: Comput Math Methods Med.

#### 2.2.1. Data Preprocessing

To fit the input to the Faster RCNN, the CT images are first preprocessed. To standardize the images, including graying out the images, uniform size, and resolution, ① CT images are mainly in black and white tones and need to be grayed out. After the grayscale operation, the number of image channels is reduced, which can effectively improve the efficiency of image processing. This study uses the PIL library method that comes with Python to implement image grayscale. ② When the scale difference between images is significant, the image features will also vary greatly, which will significantly impact the training model's speed and results. This study also uses the self-contained PIL library in Python to process the size and resolution of the images so that they match the input size of the iterative learning network.

#### 2.2.2. Dataset Construction

Based on data preprocessing, doctors who have been practicing clinical work for more than ten years at our hospital applied the Imaging Labeling system to classify and confirm CT images and label them to build the training and validation sets for deep learning networks.

According to the AO spine classification 2015, vertebral fractures are classified as type A (vertebral compression), type B (anterior-posterior distraction injury), type C (anterior-posterior rotational injury), A2 (fracture line involving both endplates but not the posterior wall of the vertebral body), A3 (vertebral fracture involving only a single endplate and involving both the posterior wall and the spinal canal), and A4 (vertebral fracture involving both upper and lower endplates and the posterior wall).

For the selected sample, the classification method proposed in this study can also deal with the presence of multiple fractures in the thoracolumbar spine, considering the practical situation where multiple different types of fractures may exist simultaneously on a single CT image.

Of the three basic types of ABC, a total of 935 thoracolumbar fracture images were selected for training and validation in this study, including 815 in the training set and 120 in the validation set, including 160 for type C, 319 for lumbar A, 48 for lumbar B, 350 for thoracic A, and 58 for thoracic B; 711 for males and 224for females; and 15 to 35 years of age, with an average of 20 years. A total of 198 thoracolumbar fracture images were selected as the test sample, of which 32 were C type, 70 were lumbar A type, 12 were lumbar B type, 80 were thoracic A type, and 15 were thoracic B type; 148 were male, and 47 were female; and the ages ranged from 17 to 36 years, with a mean of 25 years.

The article "A Classification Method for Thoracolumbar Vertebral Fractures due to Basketball Sports Injury Based on Deep Learning" was published in 2022. Journal: Comput Math Methods Med.

In the subtype classification study of type A fractures, a total of 523 images of thoracolumbar fractures were selected for training and validation, including 5489 images in the training set and 34 images in the validation set, including 46 images of type A1, 28 images of type A2, and 240 images of type A2. A3 type and A4 type were 175; 371 males and 151 females, aged 15 to 35 years old, with an average of 20 years old. 113 sheets were selected as test samples, including 15 sheets of type A1, 17 sheets of type A2, 34 sheets of type A3, and 47 sheets of type A4; 74 sheets for men and 20 sheets for women; aged 17 to 36 years old, with an average of 25 years old.

#### 2.2.3. Applying Convolutional Neural Networks to Extract Features

Faster RCNN consists of 2 modules: region proposal network (RPN) candidate frame extraction module + Fast RCNN detection module. In Faster RCNN, the training image is input to the VGG16 convolutional neural network to extract the features of the image; the RPN layer generates the candidate frames, and then, each “candidate frame” is mapped to the feature map to obtain the feature map of the region of interest; the pooling layer of the region of interest divides each candidate region into *M* × *N* blocks (whereby *M* denotes pool height, and *N* denotes pool width). The pooling layer divides each candidate region into *M* × *N* blocks (*M* denotes the pool height and *N* denotes the pool width). The maximum pooling operation is performed for each block so that the candidate regions of different sizes are transformed into feature vectors of uniform size during the feature mapping process and then fed to the next layer. The pooling layer makes the output feature map consistent with the dimensionality of the fully connected layer after it. Finally, Softmax Loss (detecting classification probability) and Smooth L1 Loss (detecting edge regression) are used for classification and regression, as shown in Figure 1.

The convolution layer is also known as the feature extraction layer. The convolutional layer contains 3 layers of convolution, pooling, and activation. To accommodate fracture image classification, this study's Faster RCNN learning model has 13 convolutional and activation layers and 4 pooling layers, as shown in Figure 2 for the specific structure.

The RPN operates as follows: a sliding scan is performed on the final convolutional feature map using a small network, and sliding window processing ensures that the regression and classification layers are associated with the entire feature space of the convolutional layer. This is then mapped to a low-dimensional vector, and finally, this low-dimensional vector is sent to the regression and classification layers to output classification diagnostics, as shown in Figure 3.

The article "A Classification Method for Thoracolumbar Vertebral Fractures due to Basketball Sports Injury Based on Deep Learning" was published in 2022. Journal: Comput Math Methods Med.

### 2.3. Evaluation Indicators

In this study, according to the classification results of the test set, the overall correct rate and kappa coefficient are used as the evaluation indexes of the overall classification effect, where the correct overall rate is the proportion of all correctly classified samples to the total samples, which is an assessment of the overall accuracy; the kappa coefficient reflects the consistency between the classification results of the classifier and the actual results. The Faster RCNN is a multiclassification network, for each class. For each category, we split it into multiple binary categories for calculation, such as for ABC-type fracture typing; when calculating the evaluation index, the problem of five categories is split into five binary categories, and the single category correct rate, sensitivity, specificity, positive predictive value, negative predictive value, and Jorden index are used as the evaluation index for the classification effect of a category, where the single category correct rate is the proportion of samples to the total samples for whether the classification is correct for a specific type. The sensitivity is the proportion of all positive cases that are correctly classified, which measures the capability of the classifier to identify positive cases; the specificity is the probability of correctly predicting the “true negative” case, which measures the ability of the model to identify negative cases; the positive predictive value is the proportion of the samples classified as positive cases that are actually positive cases. The loss value is a measure of the difference between the output of the trained model and the actual result and is related to the choice of the loss function and the number of iterations.

### 2.4. Statistical Methods

SPSS 24.0 software was used to analyze the data statistically. Correctness, sensitivity, specificity, positive predictive value, negative predictive value, Youden index, and kappa coefficient were selected for statistical analysis according to data characteristics. The test level was *α* = 0.05.

## 3. Results

### 3.1. ABC-Type Classification Test Results

The results of the classification of the ABC type are shown in Table 1. Of the 30 C-type fractures identified, 1 was not identified, 2 were incorrectly identified as thoracic A type, and 27 were correctly identified. Among the 71 lumbar type A fractures, 4 were incorrectly identified as thoracic type A, and 67 were correctly identified. Of the 12 lumbar type B fractures identified, 2 were incorrectly identified as lumbar type A and 10 were correctly identified. Of the 72 thoracic A fractures identified, 4 were not identified, 2 were incorrectly identified as lumbar A, and 66 were correctly identified. Of the 13 thoracic spine type B fractures identified, 2 were incorrectly identified as thoracic type A and 11 were correctly identified. The correct overall rate for this classification was 89.4%, with a kappa coefficient of 0.849 (*P* 0.001).  Table 2 shows the single class correct rate, sensitivity, specificity, positive predictive value, negative predictive value, and Jorden index for each category calculated from this result. Examples of successful identifications are shown in Figures 4(a) and 4(b), and examples of incorrect identifications are shown in Figures 4(c) and 4(d).  Figure 5 shows the relationship between the loss values and the number of iterations during ABC-type classification training.

The article "A Classification Method for Thoracolumbar Vertebral Fractures due to Basketball Sports Injury Based on Deep Learning" was published in 2022. Journal: Comput Math Methods Med.

### 3.2. Type A Subtype Classification Test Results

The results of the classification of type A subtypes are shown in Table 3. Of the 12 type A1 fractures, 1 was not identified, 1 was incorrectly identified as type A4, and 10 were correctly identified. Among 13 A2-type fractures, 4 were incorrectly identified as A4 type, and 9 were correctly identified. Of the 38 A3 fractures, 1 was not identified, 2 were incorrectly identified as A4, and 35 were correctly identified. Of the 41 A4 fractures, 3 were not identified, 1 was incorrectly identified as A3, and 37 were correctly identified. The correct overall rate for this classification was 87.5%, with a kappa coefficient of 0.817 (*P* < 0.001).  Table 4 shows the single class correctness, sensitivity, specificity, positive predictive value, negative predictive value, and Jorden index calculated from this result.  Figure 6 shows examples of successful and incorrect identifications.  Figure 7 shows the relationship between the loss value and the number of iterations during subtype A classification training.

## 4. Discussion

In this study, deep learning technology was applied to the classification of human thoracolumbar fractures, and a large number of CT images were screened, preprocessed, renamed, and sample annotated; after which Faster RCNN was used to learn and train the sample data of thoracolumbar fractures, establish the classification model and method of thoracolumbar fractures, and apply the CT images of human thoracolumbar fractures to test experiments.

For the classification of type ABC fractures, the overall correct classification rate of the classification model was 86.4%, with a kappa coefficient of 0.850. The sensitivity and specificity of the classification of type A fractures were higher, above 90%, for both thoracic and lumbar spine. Also, there were more unmarked samples for type A compared with type B and C. This may be caused by the bias of irregular shading in the type A dataset. Moreover, the unmarked cases are rarely found in the coronal plane and are mainly concentrated in the sagittal plane. This is because types A3 and A4 are both burst fractures with a richer fracture pattern, leading to increased difficulty in classification.

The article "A Classification Method for Thoracolumbar Vertebral Fractures due to Basketball Sports Injury Based on Deep Learning" was published in 2022. Journal: Comput Math Methods Med.

Type C ranked 2nd in the Jorden index. Of the 904 training and 35 validation images, 160 were type C, a smaller percentage than type A. The main reason for type C being misidentified is that in the coronal plane type C is so similar to type A that features characterizing type C osteochondral misalignment are only available when in the sagittal plane. Type C and type B can have similar problems in the coronal plane. In the case of similarity, the misidentification as type A is mainly due to the higher proportion of type A pictures, which obtains a more comprehensive characterization of the characterized type A fracture caused by the uneven proportion of data set types. Type C can have a higher correct rate because it is a displaced fracture morphologically more different from A and B and can be easily distinguished.

Type B fractures had the lowest Jorden index in the test, between 0.7 and 0.8, with a specificity of 100%, mainly because too few type B samples were used to train the network, even less than type C. There was an imbalance between the sample proportions, and the learning network model learned the features of type A and C fractures better; secondly, type B tends to be a fracture of the bone joint extending into the spinous portion when the fracture of the spinous is not apparent; it is easy to misidentify type B as type A.

For subtype A fracture classification, the overall correctness of the model was 85.3%, with a kappa coefficient of 0.815. The sensitivity was relatively high for types A3 and A4, exceeding 90%. The main problem with A3 and A4 identification was mutual misidentification. Type A3 fractures had only one endplate fracture, while A4 had both upper and lower endplates fractured. The distinction between A3 and A4 can only be made by whether 2 endplates are involved, and the difference between the two is slight, which is the main reason for their confusion. In addition, both A3 and A4 are burst fractures with diverse and variable fracture patterns. In a way, the amount of data in the training sample of 500 cases was insufficient, leading to unmarked A3 and A4 types.

The article "A Classification Method for Thoracolumbar Vertebral Fractures due to Basketball Sports Injury Based on Deep Learning" was published in 2022. Journal: Comput Math Methods Med.

The sensitivity of both A1 and A2 recognition is low, mainly due to the small training set of A1 and A2. Except for the unmarked cases, the false identifications are all types A3 and A4 due to the relatively large proportion of A3 and A4 in this dataset. In this study, the type ratio has been artificially balanced in the selection of images so that the number of A1 and A2 is similar and the number of A3 and A4 is similar, which will ensure a specific recognition correct rate with insufficient samples in the dataset.

This study's results show that the sensitivity of type B, type C, and two subtypes, A1 and A2, is lower than that of type A and types A3 and A4, respectively. Due to the small number of cases of these fracture types, the amount of data for these types is not enough compared to the amount of data for other types, and the learning network cannot fully extract the features of these fracture types, resulting in poorer recognition of these types. Deep learning has high requirements for dataset quality, and the acquisition of medical images is heavily dependent on clinical cases, making it difficult to establish a universal image dataset. This study found that the proportion of different types in the dataset also impacts the experimental results. Based on clinical experience, patients with A1 and A2 fracture types are themselves fewer, and some fracture cases are less distinctive, resulting in less easy identification by the machine; A3 and A4 types are more concentrated but have more fracture manifestations, resulting in the learning network not learning enough comprehensive features for correct identification. The imbalance in the proportion of dataset types can lead to the misidentification of the less represented categories as the more represented ones. The uneven distribution of the dataset due to insufficient clinical imaging data will impact the experimental results and require an increase in sample size to reduce bias in further studies.

The next issue is the number of training datasets and iterations. The ABC typing in this study used 935 training and validation sets and 10,000 iterations of learning. Before the final training, 10,000, 3,000, and 6,000 iterations were used successively, whose recognition results had a significant loss to achieve the expected results, and the number of iterations of 10,000 obtained better results. Therefore, it can be concluded that the size of the training set directly affects the classification and recognition results, which could be solved using other advanced machine learning techniques [20].

The article "A Classification Method for Thoracolumbar Vertebral Fractures due to Basketball Sports Injury Based on Deep Learning" was published in 2022. Journal: Comput Math Methods Med.

## 5. Conclusion

In summary, this study starts from the current problems faced by diagnosing spinal fractures caused by basketball injuries and introduces the latest deep learning methods for fracture diagnosis classification. The advanced thoracolumbar fracture classification method can realize the machine's autonomous fracture detection and fracture classification, which helps to shorten the time required for manual diagnosis, effectively promote high-quality medical resources, and improve the accuracy and consistency of early diagnosis of spinal fractures, thereby improving the early diagnosis of spinal fractures, efficacy of treatment of fractures.

There are still some limitations in this study: with a small sample data size, the classification accuracy of the method proposed in this research is not high, and it is easy to miss and misidentify. Future research will focus on solving the above small sample problem and achieving accurate learning for fracture patterns by changing the network structure and algorithm.

## Figures and Tables

**Figure 1:** Faster RCNN learning classification process diagram. ROI: region of interest; Feature map: feature map.

**Figure 2:** Convolutional layer specific structure.

**Figure 3:** RPN layer specific structure.

**Figure 4:** Example of ABC-type classification test results. (a) Correct identification of C fracture (sagittal). (b) Correct identification of A fracture (coronal). (c) Misidentification of lumbar A as thoracic A (sagittal). (d) Misidentification of thoracic B as lumbar B (sagittal) as lumbar type B (sagittal).

**Figure 5:** ABC-type classification loss.

**Figure 6:** Example of ABC-type classification test results. (a) Correctly identified type A3 (coronal). (b) Correctly identified type A3 (sagittal). (c) Correctly identified type A4 (coronal). (d) Correctly identified type A4 (sagittal). (e) Correctly identified A1, A4 type (sagittal). (f) Misidentified A1 type as A4 type (sagittal). (g) Misidentified A3 type as A4 type (sagittal). (h) Misidentified A4 type as A3 type (sagittal).

**Figure 7:** Type A subfractional loss.

**Table 1:** ABC-type classification test results (sheets).

Intelligent classification	Manual marking					Total
	Type C	Lumbar spine type A	Lumbar spine type B	Thoracic spine type A	Thoracic spine type B	
Type C	27	0	0	0	0	27
Lumbar spine type A	0	67	2	2	0	71
Lumbar spine type B	0	0	10	0	0	10
Thoracic spine type A	2	4	0	66	2	72
Thoracic spine type B	0	0	0	0	11	11
No identification	1	0	0	4	0	5
Total	30	71	12	72	12	197

**Table 2:** ABC typing test evaluation.

Type of fracture	Single category correct rate	Sensitivity	Specificity	Positive predictive value	Negative predictive value	Youden index
Type C	0.979	0.883	1.000	1.000	0.979	0.875
Lumbar spine type A	0.952	0.967	0.957	0.932	0.964	0.893
Lumbar spine type B	0.988	0.777	1.000	1.000	0.986	0.770
Thoracic spine type A	0.909	0.902	0.920	0.867	0.951	0.826
Thoracic spine type B	0.981	0.786	0.998	1.000	0.979	0.788

The article "A Classification Method for Thoracolumbar Vertebral Fractures due to Basketball Sports Injury Based on Deep Learning" was published in 2022. Journal: Comput Math Methods Med.

**Table 3:** Class A subtype classification test results (sheets).

Type of fracture	Single category correct rate	Sensitivity	Specificity	Positive predictive value	Negative predictive value	Youden index
Type A1	0.985	0.875	1.000	0.999	0.979	0.877
Type A2	0.947	0.940	0.958	0.919	0.964	0.896
Type A3	0.983	0.773	0.988	1.000	0.986	0.772
Type A4	0.916	0.902	0.922	0.8655	0.940	0.825

**Table 4:** Type A subtyping test evaluation.

Intelligent classification	Manual marking				Total
	Type A1	Type A2	Type A3	Type A4	
Type A1	10	0	0	0	10
Type A2	0	12	0	0	12
Type A3	0	0	35	3	38
Type A4	6	7	2	46	61
No	1	0	1	3	5
Total	17	19	38	52	126

## Data Availability

The data used to support the findings of this study are available from the corresponding author upon request.
